The article "Dysregulation of cell cycle related genes and microRNAs distinguish the low- from high-risk of prostate cancer" was retracted in 2015. Reasons: misconduct by a third party; compromised peer review.

# Dysregulation of cell cycle related genes and microRNAs distinguish the low- from high-risk of prostate cancer

**DOI:** 10.1186/s13000-014-0156-1

**Published:** 2014-09-26

**Authors:** Jiling Wen, Rongbing Li, Xiaofei Wen, Guangming Chou, Jiasun Lu, Xuelei Wang, Yongchao Jin

**Affiliations:** Department of Urology, East Hospital, Tongji University School of Medicine, Jimo Road, Shanghai, 200120 China

**Keywords:** Prostate cancer, Differentially expressed genes, MicroRNAs

## Abstract

**Background:**

Prostate cancer (PCa) is a biologically heterogeneous disease with considerable variation in clinical aggressiveness. In this study, bioinformatics was used to detect the patterns of gene expression alterations of PCa patients.

**Methods:**

The gene expression profile GSE21034 and GSE21036 were downloaded from Gene Expression Omnibus (GEO) database. Significantly changed mRNA transcripts and microRNAs were identified between subtypes with favorable (cluster 2) and unfavorable (cluster 5) prognosis by two-side unequal variances *t* test. MicroRNAs and their potential target genes were identified by TargetScan and miRTarBase, respectively. Besides, the overlapped genes between the target genes of microRNAs and mRNA transcripts were assessed by Fisher’ exact test (one side). The functional annotation was performed by DAVID, followed by construction of protein-protein interaction (PPI) network.

**Results:**

Compared to cluster 2, 1556 up-regulated and 1288 down-regulated transcripts were identified in cluster 5. Total 28 microRNAs were up-regulated and 30 microRNAs were down-regulated in cluster 5. Besides, 12 microRNAs target transcripts were significantly overlapped with down-regulated transcripts in cluster 5 with none of them was found overlapped with up-regulated transcripts. Functional annotation showed that cell cycle was the most significant function. In the PPI network, BRCA1, CDK1, TK1 and TRAF2 were hub protein of signature genes in cluster 5, and TGFBR1, SMAD2 and SMAD4 were hub proteins of signature gnens in cluster 2.

**Conclusions:**

Our findings raise the possibility that genes related with cell cycle and dysregulated miRNA at diagnosis might have clinical utility in distinguishing low- from high-risk PCa patients.

**Virtual slides:**

The virtual slide(s) for this article can be found here: http://www.diagnosticpathology.diagnomx.eu/vs/13000_2014_156

## Background

Prostate cancer (PCa) is a highly prevalent disease in older men of the western world [1]. In the US, total 241,740 men were diagnosed as PCa and 28,170 of them died for the year 2012 [2]. Although the age-adjusted rate of cancer deaths has decreased steadily in the past 10 years, PCa remains the second leading cause of cancer deaths in men after lung cancer [3]. The morbidity and mortality of PCa is mainly caused by its propensity to metastasize to other organs and tissues, such as lung, liver and bone [4,5].

The article "Dysregulation of cell cycle related genes and microRNAs distinguish the low- from high-risk of prostate cancer" was retracted in 2015. Reasons: misconduct by a third party; compromised peer review.

The clinical heterogeneity of PCa, coupled with its high prevalence, raises challenges in the management of newly diagnosed patients as well as those with metastatic disease. Genomic-based classification offers the hope of more informed clinical decision-making and may yield novel therapeutic targets. To date, several potential biomarkers including prostate cancer gene 3, methylation, human kallikrein 2, prostate-specific membrane antigen have been identified for the detection of PCa through molecular, biological, and genetic studies, but their predictive value remains to be conclusively verified [6-9].

Taylor et al. [10] reported the concordant assessment of DNA copy number, mRNA and microRNAs expression, and focused exon resequencing in prostate tumors. The copy number alteration (CNA) analysis in that study revealed two notable subgroups of primary tumors: those with minimal CNA (clusters 1–4) and those with substantial CNA (clusters 5–6) that include most of the metastatic samples. Cluster 5 and 6 are distinguished by the fact that cluster 5 tumors have genome-wide alterations, whereas those in cluster 6 primarily have 8q (NCOA2, MYC) or chromosome 7 gains. Among the tumors with minimal CNA, cluster 2 is characterized by largely unaltered genomes. Using the endpoint of time to biochemical relapse, primary tumors with generally diploid tumors in the minimally altered cluster 2 had an extremely favorable prognosis versus an extremely unfavorable prognosis for the highly altered cluster 5 tumors. However, the detailed genomic differences between cluster 2 with favorable prognosis and cluster 5 with extremely unfavorable prognosis are remaining unclear.

To reveal the potential genes and microRNAs which might have clinical utility in distinguishing low- from high-risk disease, we investigated the gene and microRNAs expression profile between cluster 2 and cluster 5 PCa patients in the present study.

## Methods

### Microarray datasets

Normalized mRNA and microRNAs expression profile data (GSE21034 and GSE21036) were downloaded from Gene Expression Omnibus (GEO). Only mRNA transcripts with Reference Sequence (Refseq) identifiers prefixed with “NM_” were retained. MicroRNAs profiling data were available for 8 (classified as cluster 5) and 25 PCa patients (classified as cluster 2), while mRNA profiling data were available for 13 (classified as cluster 5) and 34 PCa patients (classified as cluster 2). The ethical committee of Memorial Sloan-Kettering Cancer Center Institutional Review Board approved the study protocol and informed consent was obtained from all the patients.

The article "Dysregulation of cell cycle related genes and microRNAs distinguish the low- from high-risk of prostate cancer" was retracted in 2015. Reasons: misconduct by a third party; compromised peer review.

### Identification of differentially expressed mRNA transcripts and microRNAs

Two-side unequal variances *t* test was used to identify the differentially expressed mRNA transcripts between cluster 2 and cluster 5. q value [11] is a well suited measure of significance for genomewide tests with an extension of a quantity called the “false discovery rate” (FDR). q value < 0.05 was selected as cutoff. Significantly changed mRNA transcripts were submitted to the online tool Database for Annotation, Visualization, and Integrated Discovery (DAVID) for functional annotation and molecular signatures database (MSigDB) for finding out potential links with published gene expression signature. For microRNAs analysis, two-side unequal variance *t* test was performed with the threshold of P < 0.05.

### Identification of microRNA and their potential target gene

TargetScan [12] can predict biological targets of miRNAs by searching for the presence of conserved 8mer and 7mer sites that match the seed region of each miRNA. The miRTarBase [13] is a database which contains experimentally validated microRNA-target interactions. Target genes were downloaded from TargetScan 6.2 and experimentally validated target genes from miRTarBase (version 3.5). Fisher’ exact test [14] (one side) was used to assess the statistical significance of the overlapped genes between the target genes of microRNAs and mRNA transcripts.

### Construction of protein-protein interaction (PPI) network

Most proteins perform their functions through interactions and high-quality interaction networks can provide key insights into fundamental topological and biological properties of cellular systems. Thus, the PPI data were downloaded from HINT [15] database for construction of PPI network of significantly changed signature genes. Refseq mRNA identifiers were mapped to EntrezGene identifiers and extracted the interactions between significantly changed signature genes. Proteins with at least ten interactions were considered as hubs in the present study.

## Results

### Identification of significantly altered transcripts between cluster 2 and cluster 5

Compared with cluster 2, 1556 transcripts were found up-regulated and 1288 transcripts were down-regulated in cluster 5. Functional annotation analysis revealed that Cluster 5 signature genes were mainly enriched in the cell cycle and proliferation pathways, while cluster 2 signature genes were enriched in the pathways of response to stimulus, like steroid hormone. MSigDB investigation showed that these PCa subtype signature was correlated with many published gene signature. The most interesting finding was that the down-regulated genes in PC3 cell after knockdown of EZH2 by RNAi were significantly overlapped with the cluster 5 gene signature, and up-regulated genes were significantly overlapped with the cluster 2 gene signature. Compared to cluster 2, two mRNA transcripts (NM_004456, NM_152998) of EZH2 were significantly up-regulated in cluster 5.

The article "Dysregulation of cell cycle related genes and microRNAs distinguish the low- from high-risk of prostate cancer" was retracted in 2015. Reasons: misconduct by a third party; compromised peer review.

### Identification of dysregulated microRNAs and their potential target gene

Compared with cluster 2, 28 microRNAs were up-regulated and 30 microRNAs were down-regulated in cluster 5 (Table 1). Besides, 12 microRNAs target transcripts were significantly overlapped with down-regulated transcripts in cluster 5. However, no microRNA target transcript was found overlapped with up-regulated transcripts in cluster 5 (Table 2).

**Table 1:** **MicroRNAs that significantly changed in cluster 2 and 5**

	**MicroRNAs**	**Fold-change**	**P-value**	**Chromosome region**
Up-regulated				
	hsa-miR-151-3p	1.08	2.5 E-2	8
	hsa-miR-1237	1.33	8.8 E-3	11
	hsa-miR-548c-3p	1.63	2.6 E-2	12
	hsa-miR-1228	1.14	1.8 E-2	12
	hsa-miR-130b	1.13	9.2 E-3	22
	hsa-miR-210	1.17	3.5 E-2	11p15.5
	hsa-miR-141	1.07	1.18 E-2	12p13.31
	hsa-miR-19b-1*	1.30	4.06 E-2	13q31.3
	hsa-miR-627	1.23	2.65 E-2	15q15.1
	hsa-miR-1225-3p	1.15	4.85 E-2	16p13.3
	hsa-miR-33b	2.10	4.08 E-3	17p11.2
	hsa-miR-423-3p	1.22	2.15 E-2	17q11.2
	hsa-miR-423-5p	1.09	2.26 E-2	17q11.2
	hsa-miR-636	1.21	1.38 E-2	17q25.1
	hsa-let-7a*	1.50	9.55 E-3	22q13.31
	hsa-miR-191*	1.33	3.78 E-4	3p21.31
	hsa-miR-425*	1.26	6.50 E-3	3p21.31
	hsa-miR-16-2*	1.18	3.39 E-2	3q25.33
	hsa-miR-148a*	1.26	2.59 E-2	7p15.2
	hsa-miR-93	1.08	2.32 E-2	7q22.1
	hsa-miR-106b	1.06	4.87 E-2	7q22.1
	hsa-miR-335*	1.39	3.20 E-2	7q32.2
	hsa-miR-182	1.20	8.72 E-3	7q32.2
	hsa-miR-30d*	1.27	2.81 E-2	8q24.22
	hsa-miR-30d	1.07	1.99 E-2	8q24.22
	hsa-miR-491-5p	1.45	2.64 E-2	9p21.3
	hsa-miR-602	1.24	1.13 E-2	9q34.3
	hsa-miR-542-5p	1.20	2.15 E-2	Xq26.3
Down-regulated				
	hsa-miR-130a	0.87	2.70 E-2	11q12.1
	hsa-miR-100	0.85	2.40 E-2	11q24.1
	hsa-miR-125b	0.90	3.80 E-2	11q24.1,21q21.1
	hsa-miR-136*	0.85	2.90 E-2	14q32.2
	hsa-miR-495	0.82	4.48 E-2	14q32.31
	hsa-miR-132	0.88	1.03 E-2	17p13.3
	hsa-miR-132*	0.89	1.70 E-2	17p13.3
	hsa-miR-152	0.89	3.24 E-2	17q21.32
	hsa-miR-338-3p	0.82	5.61 E-4	17q25.3
	hsa-miR-133a	0.71	3.41 E-3	18q11.2,20q13.33
	hsa-miR-30e*	0.89	3.59 E-2	1p34.2
	hsa-miR-30c	0.90	2.41 E-2	1p34.2,6q13
	hsa-miR-205	0.63	4.50 E-2	1q32.2
	hsa-miR-499-5p	0.83	2.61 E-2	20q11.22
	hsa-miR-1	0.69	3.76 E-3	20q13.33
	hsa-miR-218	0.83	1.79 E-2	4p15.31,5q34
	hsa-miR-145*	0.74	1.01 E-2	5q32
	hsa-miR-143	0.78	1.64 E-2	5q32
	hsa-miR-143*	0.80	1.24 E-2	5q32
	hsa-miR-145	0.86	2.43 E-2	5q32
	hsa-miR-378*	0.93	2.50 E-2	5q32
	hsa-miR-133b	0.77	6.36 E-3	6p12.2
	hsa-miR-204	0.72	1.79 E-2	9q21.12
	hsa-miR-24-1*	0.79	7.48 E-3	9q22.32
	hsa-miR-27b	0.88	1.29 E-2	9q22.32
	hsa-miR-23b	0.88	2.56 E-2	9q22.32
	hsa-miR-455-5p	0.76	5.74 E-3	9q32
	hsa-miR-455-3p	0.80	2.85 E-2	9q32
	hsa-miR-221*	0.67	670 E-4	Xp11.3
	hsa-miR-221	0.80	4.19 E-3	Xp11.3
	hsa-miR-223	0.90	2.59 E-2	Xq12

“*” stands for the miRNA which is expressed at low levels.

The article "Dysregulation of cell cycle related genes and microRNAs distinguish the low- from high-risk of prostate cancer" was retracted in 2015. Reasons: misconduct by a third party; compromised peer review.

**Table 2:** **TargetScan target transcripts of microRNAs that up-regulated in cluster 5 significantly overlapped with mRNA transcripts that down-regulated in cluster 5 compared to cluster 2**

	**Number of targets**	**Number of overlapped targets**	**p-value**
hsa-miR-548c-3p	2611	288	3.62E-38
hsa-miR-30d	1773	195	4.37E-25
hsa-miR-130b	1205	151	5.33E-25
hsa-miR-93	1583	153	1.18E-14
hsa-miR-106b	1583	153	1.18E-14
hsa-miR-33b	544	69	3.44E-12
hsa-miR-141	996	102	1.66E-11
hsa-miR-636	874	92	3.97E-11
hsa-miR-182	1494	131	8.35E-10
hsa-miR-1228	274	34	1.74E-06
hsa-miR-602	33	7	1.19 E-3
hsa-miR-151-3p	145	16	3.12 E-3

Note: Fisher’s exact test was applied to assess the statistical significance and only those with p-value < 0.005 were shown.

### PPI network analysis

The results of PPI network analysis showed that there were 46 nodes and 46 edges in cluster 5 (Figure 1). Meanwhile, total 27 nodes and 34 edges were in cluster 2 (Figure 2). Proteins with at least ten interactions were considered as hubs. The results revealed that BRCA1, CDK1, TK1 and TRAF2 were hub protein of signature genes in cluster 5, and TGFBR1, SMAD2 and SMAD4 were hub proteins of signature gnens in cluster 2.

**Figure 1:** **Protein-protein interactions in cluster 5 signature genes.** Yellow nodes are those interacted with androgen receptor. Protein-protein interactions were downloaded from database HINT which removes low-quality/erroneous interactions by both systematically and manually filtering.

**Figure 2:** **Protein-protein interactions in cluster 2 signature genes.** Protein-protein interactions were downloaded from database HINT which removes low-quality/erroneous interactions by both systematically and manually filtering.

## Discussion

The clinical heterogeneity of PCa, coupled with its high prevalence, raises challenges in the management of newly diagnosed patients as well as those with metastatic disease. Genomic-based classification offers the hope of more informed clinical decision and may yield novel therapeutic targets. In this bio-information analysis, we found that cell cycle was selected as the most significant pathway. The androgen receptors (AR) related genes, such as CDK1 and BRCA1 might play important roles in the development of PCa.

The article "Dysregulation of cell cycle related genes and microRNAs distinguish the low- from high-risk of prostate cancer" was retracted in 2015. Reasons: misconduct by a third party; compromised peer review.

### Transcriptions in cluster 5 were associated with EZH2-mediated regulation

EZH2 encodes a member of the Polycomb-group (PcG) family which involved in maintaining the transcriptional repressive state of genes over successive cell generations. Xu K et al. [16] have found that the oncogenic function of EZH2 in cells of castration-resistant PCa is independent of its role as a transcriptional repressor. Instead, it involves the ability of EZH2 to act as a coactivator for critical transcription factors including AR. Phosphorylation of EZH2 and an intact methyltransferase domain were required for this functional switch. In the present study the transcriptions in cluster 5 were overlapped with those down-regulated genes after knockdown of EZH2. Indeed, two mRNA transcripts (NM_004456, NM_152998) of EZH2 were significantly up-regulated in cluster 5 PCa compared to cluster 2. Our finding of PCa subtype gene signature was associated with EZH2-mediated regulation which further addressed the important role of EZH2 in the progress of PCa.

### The up-regulated genes which were related to cell cycle in cluster 5 might have prognostic value

Functional annotation in the present study showed that Cluster 5 up-regulated signature genes were mainly associated with cell cycle. Proper regulation of the cell division cycle is crucial to the growth and development of all organisms. Actually, some cell cycle progression (CCP) genes have been identified as having RNA expression levels that oscillated as cells progressed through various stages of the cell cycle [17]. Cell cycle-regulated transcripts of genes involved in fundamental processes such as DNA replication and chromosome segregation seem to be more highly expressed in proliferative tumors simply because they contain more cycling cells. Mandal et al. [18] suggested that there was a positive association of cyclin D1AA genotype and diplotype analysis of Fas G670A and G1377A (G-A) which was associated with CaP risk by influencing the pathophysiology of CaP. Cuzick et al. [19] found that the cell cycle progression signature was a highly significant predictor of outcome in both cohorts of PCa patients. Since the expression levels of CCP genes probably reflect fundamental aspects of tumour biology, we reasoned that the up-regulated genes related with cell cycle in the present study might also be useful in PCa.

### MicroRNAs could play regulatory roles of PCa subtype gene signature

In the present study, miR-1 was found significantly up-regulated in cluster 5 PCa. Kojima et al. found that the expression levels of miR-1 and miR-133a were significantly down-regulated in PCa compared with non-PCa tissues [20]. Restoration of miR-1 or miR-133a in PC3 and DU145 cells revealed significant inhibition of proliferation, migration, and invasion. They further suggest that miR-1 and miR-133 could be tumor suppressors by targeting purine nucleoside phosphorylase (PNP). Other microRNAs also has close relationship with PCa, for example, loss of microRNA-126 has been reported to play a positive role in the progression of PCa [21]. Meanwhile, we also found that predicted targets of other up-regulated microRNAs could significantly overlap with down-regulated genes in cluster 5 PCa. The roles of these microRNAs in PCa might worth further investigating according to the previous studies [22-24].

The article "Dysregulation of cell cycle related genes and microRNAs distinguish the low- from high-risk of prostate cancer" was retracted in 2015. Reasons: misconduct by a third party; compromised peer review.

### BRCA1 and CDK1, both interacted with AR were hub proteins of cluster 5

Genetic factor has been considered to be critical in the development and progression of PCa. Aldo-keto reductase family 1 member C3 (AKR1C3) has been found to serve as a hopeful biomarker and is closely related to the progression of PCa [25]. In the present study, we found *BRCA1* and *CDK1* were strong related to PCa. The expression of AR is maintained throughout PCa progression, and the majority of androgen-independent or hormone refractory PCa express AR. Similarly, alterations in the relative expression of AR coregulators have been found to occur with PCa progression and may contribute to differences in AR ligand specificity or transcriptional activity [26]. Inhibiting AR signaling remains one of the most common and effective systemic methods to treat PCa. BRCA1 might function as an AR coregulator and directly modulate AR signaling [27]. Yeh S et al. report that BRCA1 interacts with androgen receptor and enhances AR target genes, such as p21 (WAF1/CIP1) that may result in the increase of androgen-induced cell death in PCa cells [28]. Another hub protein CDK1 was also found to be significantly expressed in “androgen-independent” PCa which relapse subsequent to androgen-deprivation therapy. It was suggested that AR is active and seems to be stabilized by low level of androgen in such PCa and treatment with roscovitine, a Cdk inhibitor, could abrogate responses to low levels of androgen in the androgen-independent PCa cell line [29].

Our analysis also addresses the important role of TGF-beta signaling in cluster 2 PCa. Combined with our finding, investigation of the roles of TGFBR1 and SMAD4 in PCa could be of great value. However, there were still some limitations in this study. A further investigation in cluster 2 and 5 related to PCa is needed.

## Conclusion

In summary, our findings raise the possibility that genes related with cell cycle and dysregulated miRNA at diagnosis might have clinical utility in distinguishing low- from high-risk PCa patients. However, as our results were based on microarray data derived from a small sample size, further experimental validation is needed.

The article "Dysregulation of cell cycle related genes and microRNAs distinguish the low- from high-risk of prostate cancer" was retracted in 2015. Reasons: misconduct by a third party; compromised peer review.

## References

[1] Chan JM, Jou RM, Carroll PR (2004). The relative impact and future burden of prostate cancer in the United States. J Urol.

[2] Siegel R, Naishadham D, Jemal A (2012). Cancer statistics, 2012. CA Cancer J Clin.

[3] Shen MM, Abate-Shen C (2010). Molecular genetics of prostate cancer: new prospects for old challenges. Genes Dev.

[4] Berezikov E, Guryev V, Van De Belt J, Wienholds E, Plasterk RH, Cuppen E (2005). Phylogenetic shadowing and computational identification of human microRNA genes. Cell.

[5] Logothetis CJ, Lin SH (2005). Osteoblasts in prostate cancer metastasis to bone. Nat Rev Cancer.

[6] Nogueira L, Corradi R, Eastham JA (2010). Other biomarkers for detecting prostate cancer. BJU Int.

[7] Hoque MO, Kim MS, Ostrow KL, Liu J, Wisman GB, Park HL, Poeta ML, Jeronimo C, Henrique R, Lendvai A, Schuuring E, Begum S, Rosenbaum E, Ongenaert M, Yamashita K, Califano J, Westra W, Van Der Zee AG, Van Criekinge W, Sidransky D (2008). Genome-wide promoter analysis uncovers portions of the cancer methylome. Cancer Res.

[8] Schilling D, De Reijke T, Tombal B, De La Taille A, Hennenlotter J, Stenzl A (2010). The Prostate Cancer gene 3 assay: indications for use in clinical practice. BJU Int.

[9] Hoque MO (2009). DNA methylation changes in prostate cancer: current developments and future clinical implementation. Expert Rev Mol Diagn.

[10] Taylor BS, Schultz N, Hieronymus H, Gopalan A, Xiao Y, Carver BS, Arora VK, Kaushik P, Cerami E, Reva B, Antipin Y, Mitsiades N, Landers T, Dolgalev I, Major JE, Wilson M, Socci ND, Lash AE, Heguy A, Eastham JA, Scher HI, Reuter VE, Scardino PT, Sander C, Sawyers CL, Gerald WL (2010). Integrative genomic profiling of human prostate cancer. Cancer Cell.

[11] Storey JD, Tibshirani R (2003). Statistical significance for genomewide studies. Proc Natl Acad Sci U S A.

[12] Friedman RC, Farh KK, Burge CB, Bartel DP (2009). Most mammalian mRNAs are conserved targets of microRNAs. Genome Res.

[13] Hsu SD, Lin FM, Wu WY, Liang C, Huang WC, Chan WL, Tsai WT, Chen GZ, Lee CJ, Chiu CM, Chien CH, Wu MC, Huang CY, Tsou AP, Huang HD (2011). miRTarBase: a database curates experimentally validated microRNA-target interactions. Nucleic Acids Res.

[14] Daya S (2002). Fisher exact test. Evid Based Obstet Gynecol.

[15] Das J, Yu H (2012). HINT: high-quality protein interactomes and their applications in understanding human disease. BMC Syst Biol.

[16] Xu K, Wu ZJ, Groner AC, He HH, Cai C, Lis RT, Wu X, Stack EC, Loda M, Liu T, Xu H, Cato L, Thornton JE, Gregory RI, Morrissey C, Vessella RL, Montironi R, Magi-Galluzzi C, Kantoff PW, Balk SP, Liu XS, Brown M (2012). EZH2 oncogenic activity in castration-resistant prostate cancer cells is Polycomb-independent. Science.

The article "Dysregulation of cell cycle related genes and microRNAs distinguish the low- from high-risk of prostate cancer" was retracted in 2015. Reasons: misconduct by a third party; compromised peer review.

[17] Whitfield ML, Sherlock G, Saldanha AJ, Murray JI, Ball CA, Alexander KE, Matese JC, Perou CM, Hurt MM, Brown PO, Botstein D (2002). Identification of genes periodically expressed in the human cell cycle and their expression in tumors. Mol Biol Cell.

[18] Mandal RK, Mittal RD (2010). Are cell cycle and apoptosis genes associated with prostate cancer risk in North Indian population?. Urol Oncol.

[19] Cuzick J, Swanson GP, Fisher G, Brothman AR, Berney DM, Reid JE, Mesher D, Speights VO, Stankiewicz E, Foster CS, Moller H, Scardino P, Warren JD, Park J, Younus A, Flake DD, Wagner S, Gutin A, Lanchbury JS, Stone S (2011). Prognostic value of an RNA expression signature derived from cell cycle proliferation genes in patients with prostate cancer: a retrospective study. Lancet Oncol.

[20] Kojima S, Chiyomaru T, Kawakami K, Yoshino H, Enokida H, Nohata N, Fuse M, Ichikawa T, Naya Y, Nakagawa M, Seki N (2012). Tumour suppressors miR-1 and miR-133a target the oncogenic function of purine nucleoside phosphorylase (PNP) in prostate cancer. Br J Cancer.

[21] Sun X, Liu Z, Yang Z, Xiao L, Wang F, He Y, Su P, Wang J, Jing B (2013). Association of microRNA-126 expression with clinicopathological features and the risk of biochemical recurrence in prostate cancer patients undergoing radical prostatectomy. Diagn Pathol.

[22] Fang L, Deng Z, Shatseva T, Yang J, Peng C, Du WW, Yee AJ, Ang LC, He C, Shan SW, Yang BB (2011). MicroRNA miR-93 promotes tumor growth and angiogenesis by targeting integrin-beta8. Oncogene.

[23] Li Y, Tan W, Neo TW, Aung MO, Wasser S, Lim SG, Tan TM (2009). Role of the miR-106b-25 microRNA cluster in hepatocellular carcinoma. Cancer Sci.

[24] Yang IP, Tsai HL, Hou MF, Chen KC, Tsai PC, Huang SW, Chou WW, Wang JY, Juo SH (2012). MicroRNA-93 inhibits tumor growth and early relapse of human colorectal cancer by affecting genes involved in the cell cycle. Carcinogenesis.

[25] Tian Y, Zhao L, Zhang H, Liu X, Zhao X, Li Y, Li J (2014). AKR1C3 overexpression may serve as a promising biomarker for prostate cancer progression. Diagn Pathol.

[26] Heinlein CA, Chang C (2004). Androgen receptor in prostate cancer. Endocr Rev.

[27] Park JJ, Irvine RA, Buchanan G, Koh SS, Park JM, Tilley WD, Stallcup MR, Press MF, Coetzee GA (2000). Breast cancer susceptibility gene 1 (BRCAI) is a coactivator of the androgen receptor. Cancer Res.

[28] Yeh S, Hu YC, Rahman M, Lin HK, Hsu CL, Ting HJ, Kang HY, Chang C (2000). Increase of androgen-induced cell death and androgen receptor transactivation by BRCA1 in prostate cancer cells. Proc Natl Acad Sci U S A.

The article "Dysregulation of cell cycle related genes and microRNAs distinguish the low- from high-risk of prostate cancer" was retracted in 2015. Reasons: misconduct by a third party; compromised peer review.

[29] Chen S, Xu Y, Yuan X, Bubley GJ, Balk SP (2006). Androgen receptor phosphorylation and stabilization in prostate cancer by cyclin-dependent kinase 1. Proc Natl Acad Sci U S A.

